# Exploration and Practice of the Relationship between College Students' Learning Adaptation and Mental Health under the Information-Based Teaching Environment of Potential Profile Analysis

**DOI:** 10.1155/2023/2256741

**Published:** 2023-02-04

**Authors:** Hongmei Zhu

**Affiliations:** Xi'an Peihua University, 710125 Xi'an, China

## Abstract

In order to further investigate and understand the relationship between college students' learning adaptation process and mental health in the learning process under the information-based teaching environment, this paper makes a questionnaire survey on college students' learning adaptation and mental health and selects 408 college students as the research object. The results show that the potential profile analysis shows that with the development of network and informatization, the learning adaptability of college students can be divided into four types: troubled group (accounting for 7.598%), marginal adaptive group (accounting for 42.892%), maladaptive group (accounting for 4.167%), and good adaptive group (accounting for 45.343%). The mental health level of the latter two is better, and the mental health level of the first two is worse. Students who do not adapt to learning and students who adapt well show common characteristics. Most of them are only children, and their parents have a high level of education. This kind of family often has good material conditions and loose family atmosphere, which will also form a protective mechanism for students' mental health, making students have good self-acceptance ability and good mental health level.

## 1. Introduction

The rapid development of network and information technology has promoted the development of many industries, especially the rapid development of information technology, which provides more technical choices and mode innovation drivers for the improvement of modern teaching methods and teaching quality. In the information-based teaching environment, students' learning process is no longer limited by the “time and space” of traditional education, and information technology can provide students with more personalized learning methods and learning contents. Compared with traditional face-to-face teaching and classroom teaching, the transformation of teaching methods will also require students to constantly adjust their learning methods. Teachers need to change, and students also need to change [1]. However, the level of students' learning adaptability directly affects the learning effect. Some students will have maladjustment in the face of the environmental changes brought by the information environment, while some students will have strong interest in learning and can adapt well due to the novel learning methods, and different adaptation results will even affect students' mental health and indirectly affect their learning status, which is also the focus of this study.

## 2. Literature Review

Some scholars believe that learning adaptability includes not only students' learning potential but also students' learning motivation, clear learning purpose, actions taken to meet academic requirements, and general satisfaction with the learning environment [2]. The expression of the concept of learning adaptation, that is, learning adaptability, refers to the tendency of individuals to overcome difficulties and achieve better learning results, that is, learning adaptability. Its main factors include learning attitude, learning technology, learning environment, and physical and mental health. At the same time, some scholars have defined learning adaptation. For example, Kelzang and Lhendup believe that learning adaptability refers to the ability tendency of students to adjust themselves to the learning environment in the learning process [3]. Xiao believes that learning adaptability is “when the learning environment, learning objects, and contents around individuals change, individuals take the initiative to overcome difficulties and change themselves in order to avoid the decline of learning efficiency, so as to achieve good learning efficiency” [4]. Kim et al. define learning adaptability as the ability of individuals to actively adjust their learning motivation and behavior, improve their learning ability, coordinate their learning psychology and behavior with the changing learning conditions, and achieve good learning achievements according to the changes of internal and external learning conditions and their own learning needs [5]. Jeong believes that learning adaptability is the psychological ability of individuals to actively react to the surrounding environment with certain behaviors and actions in the process of interaction between individuals and learning environment [6]. Mahasneh believes that learning adaptation is a psychological and behavioral process in which the subject tries to adjust himself according to the environment and learning needs, so as to achieve a balance with the learning environment. Chinese scholars have put forward their own different views and views on the concept of learning adaptation from their respective perspectives [7].

In view of the unique characteristics of Chinese college students' learning adaptability, some scholars have developed a scale suitable for measuring Chinese college students' learning adaptability. For example, based on the “learning adaptability test (middle school version),” the “college students' learning adaptability questionnaire” is compiled according to the age and learning characteristics of college students. On the basis of previous studies, a set of learning adaptability scale for college students is compiled. The questionnaire is divided into five dimensions: learning motivation adaptation, learning ability adaptation, learning environment adaptation, education style adaptation, and physical and mental health adaptation. There are 50 items in this questionnaire. The three-level scoring method is adopted. The higher the score, the better the learning adaptability. The content of the questionnaire includes two dimensions of learning motivation and learning adaptive learning behavior, as well as eight factors such as professional interest, autonomous learning, stress response, method application, help-seeking behavior, environmental choice, information utilization, and knowledge application, with a full score of five points [8, 9].

At present, the research on the learning adaptability of college students in China is still in the exploratory stage compared with the research on the learning adaptability of primary and secondary school students. The research on college students mostly focuses on the investigation and research on the learning adaptability of college freshmen. The existing literature shows that the research content of college students' learning adaptability in China also focuses on two aspects. One is the discussion of the factors affecting college students' learning adaptability. The other is that Chinese scholars have compiled some learning adaptability questionnaires suitable for Chinese college students according to their own characteristics. Scholars in China have conducted some investigation and research on the factors affecting college students' learning adaptability, as shown in Figure 1, which shows the common confusion of college students [10]. Through the investigation, it is found that college students' learning adaptability is mainly affected by many factors, such as students' own cognitive evaluation, personality characteristics, school environment, family education methods, and social support. In the aspect of cognitive evaluation, this paper studies the relationship between higher vocational college students' self-concept, coping style, and learning adaptability. The conclusion is that the total score of self-concept is significantly negatively correlated with the overall learning adaptation score, and the mature coping style is highly significantly positively correlated with the overall learning adaptation. Immature coping style has a very significant negative correlation with overall learning adaptation [11]. Some scholars have concluded that there is a close relationship between self-harmony and learning adaptability of normal college students. The research shows that there is a significant positive correlation between college students' learning adaptability and learning self-efficacy and the total score of career commitment [12].

## 3. Bayesian Analysis of Latent Variable Model under Random Effect

### 3.1. Random Effect Model

The random effect model is as follows:

(1) $$\begin{array}{c} y_{i}=x_{i}\beta +u_{i}+\varepsilon_{i},\;i=1,\ldots ,n\text{,} \end{array}$$

where

(2) $$\begin{array}{c} \beta ={\left(\beta_{1},\beta_{2},\ldots ,\beta_{q}\right)}^{T}\text{,} \end{array}$$

and *y*_*i*_, *x*_*i*_ are datasets, which are recorded as follows:

(3) $$\begin{array}{c} Y={\left(y_{1},y_{2},\ldots ,y_{n}\right)}^{T}\text{,} \end{array}$$

(4) $$\begin{array}{c} x_{i}=\left(1,x_{i1},x_{i2},\ldots ,x_{iq}\right)\text{.} \end{array}$$

Generally, it follows the normal distribution with mean value of 0 and standard deviation of *σ*_*u*_. In mean regression, it is generally assumed that the error term *ε*_*i*_ follows the error term with mean value of 0 and variance of *σ*_*ε*_^2^. Here, we consider quantile regression, so it is assumed that *ε*_*i*_ follows the Laplace distribution with unknown parameter of 0 and scale parameter of *σ*, that is,

(5) $$\begin{array}{c} \varepsilon_{i}∼\text{ALD}\left[0,\sigma \right]\text{.} \end{array}$$

Its density function is as follows:

(6) $$\begin{array}{c} f_{p}\left(\varepsilon_{i};p,\sigma \right)=\frac{p\left(1-p\right)}{\sigma }\exp\;\left\{-\rho_{p}\left(\varepsilon_{i}\right)\right\}\text{,} \end{array}$$

where the form of 0 < *p* < 1; *ρ*_*p*_(*ε*_*i*_) is as follows:

(7) $$\begin{array}{c} \rho_{p}\left(\varepsilon_{i}\right)=\frac{\left|\varepsilon_{i}\right|+\left(2p-1\right)\varepsilon_{i}}{2\sigma }\text{.} \end{array}$$

Then, the likelihood function of the random effect model can be written as

(8) $$\begin{array}{c} L\left(\left.\theta \right|Y,X\right)=\frac{p^{n}{\left(1-p\right)}^{2}}{\sigma^{n}}\exp\;\left\{-\overset{n}{\underset{i}{\sum }}\rho_{p}\left(\frac{y_{i}-x_{i}\beta -u_{i}}{\sigma }\right)\right\}\text{.} \end{array}$$

This method needs to extract samples from a posteriori distribution [*θ*|*Y*, *X*] and then obtain an empirical distribution close to the real distribution according to the samples, which can characterize the characteristics of a posteriori distribution.

Assume that the a priori distribution of *β* is as follows:

(9) $$\begin{array}{c} \beta ∼N\left[b,V\sigma \right]\text{,} \end{array}$$

where *b* is the column vector of *q* dimension; when the observation values *Y* and *X* are given, the diagonal matrix of order *q* + 1 of formula *V* is as follows:

(10) $$\begin{array}{c} p\left(\left.\beta ,Y\right|U,X,\sigma \right)=L\left(\left.\theta \right|Y,X\right)p\left(\beta \right)=p\left(\beta \right)\left(\left.\beta \right|Y,U,X,\sigma \right)p\left(Y\right)\text{.} \end{array}$$

The posterior distribution of *β* is obtained. If the prior and posterior distributions obey the same type of distribution, this prior distribution is called conjugate prior distribution. Assume a priori distribution of *U*:

(11) $$\begin{array}{c} U∼N\left[b_{u},I\sigma_{u}^{2}\right]\text{,} \end{array}$$

where the column vector of *n* dimension of formula *b*_*u*_ and the unit diagonal matrix of order *n* of formula *I* are composed of conditional distribution:

(12) $$\begin{array}{c} p\left(\left.U,Y\right|\beta ,X,\sigma \right)=L\left(\left.\theta \right|Y,X\right)p\left(U\right)=p\left(U\right)\left(\left.U\right|Y,\beta ,X,\sigma \right)p\left(Y\right)\text{.} \end{array}$$

After obtaining the prior distribution of *U*, there is the following process:

(13) $$\begin{array}{c} p\left(\left.U,Y\right|\beta ,X,\sigma \right)\propto L\left(\left.\theta \right|Y,X\right)p\left(U\right)\propto {\left(\frac{p\left(1-p\right)}{\sigma }\right)}^{n}\;\exp\;\left\{-\underset{i}{\sum }\rho_{p}\left(\frac{y_{i}-x_{i}\beta -u_{i}}{\sigma }\right)\right\}\text{,}\\ {\left|I\sigma_{u}^{2}\right|}^{-1/2}\;\exp\;\left\{-\frac{1}{2}{\left(U-b_{u}\right)}^{T}{\left(I\sigma \right)}^{-1}\left(U-b_{u}\right)\right\}\text{,}\\ \propto {\left(p\left(1-p\right)\right)}^{n}\sigma^{-n}\sigma_{u}^{-n}\exp\;\left\{-\underset{i}{\sum }\rho_{p}\left(\frac{y_{i}-x_{i}\beta -u_{i}}{\sigma }\right)-\frac{1}{2}{\left(U-b_{u}\right)}^{T}{\left(I\sigma_{u}^{2}\right)}^{-1}\left(U-b_{u}\right)\right\}\text{.} \end{array}$$

Suppose the conjugate a priori distribution of *σ*_*u*_^−2^ is as follows:

(14) $$\begin{array}{c} \sigma_{u}^{-2}∼\text{Gamma}\left[a_{1},r_{1}\right]\text{,} \end{array}$$

where *a*_1_, *r*_1_ are superparameters, which can be obtained from the conditional distribution:

(15) $$\begin{array}{c} p\left(\left.U,\sigma_{u}^{-2}\right|Y\right)=p\left(\left.\sigma_{u}^{-2}\right|U,Y\right)p\left(U\right)\propto p\left(\left.U\right|Y,\sigma_{u}^{-2}\right)p\left(\sigma_{u}^{-2}\right)\text{.} \end{array}$$

If the hyperparameters in the conjugate a priori distribution are unknown, they should be regarded as unknown parameters with a priori distribution. However, these prior distributions also have their own superparameters, so it will be difficult to extract samples. Therefore, for the convenience of research, the hyperparameters in the conjugate a priori distribution are set to known values.

The simulation of the random effect model is as follows:

(16) $$\begin{array}{c} y_{i}=0.5+0.7x_{i1}+0.7x_{i1}+0.7x_{i1}+0.7x_{i1}+u_{i}+\varepsilon_{i},i=1,\ldots ,n\text{.} \end{array}$$

Assumptions:

(17) $$\begin{array}{c} b={\left(2,\ldots ,2\right)}_{\left(q+1\right)\times 1}^{T}\text{.} \end{array}$$

Adiagonal matrix in which the diagonal elements of the formula *V* are 0.5 and *q* + 1 dimensions.

(18) $$\begin{array}{c} b_{u}={\left(2,\ldots ,2\right)}_{\left(n+1\right)}^{T}\text{.} \end{array}$$

*I* is an n-order unit matrix, and *σ*_*u*_=0.5. First, 50 sets of simulation datasets with a sample size of *n* = 100 are produced. In this example, we need to estimate *β*, *σ*, *U*, *σ*_*u*_, iterate 10000 times, and do 50 repeated calculations. The EPSR values of the parameters are close to 1, which are 0.968, 0.984, 0.975, and 0.989, respectively, indicating that the simulation process converges. Therefore, the first 9000 times are discarded and the last 1000 times are taken as the simulation results. Figures 2–5 represent the straight line diagram under different quantiles corresponding to different beta values.

Then, 50 groups of simulation datasets with sample size of *n* = 30 and 50100 are generated, and 50 repeated calculations are made, respectively. Assuming *q* = 4, the calculation model is iterated 10000 times each time, the first 9000 times are discarded, and the last 1000 times are taken as the simulation results. Considering the difference of samples and the deviation of calculated estimates, the root mean square between the actual value and the corresponding estimated value is defined as follows:

(19) $$\begin{array}{c} \theta \left(k\right)={\left\{\frac{1}{50}\overset{50}{\underset{d}{\sum }}{\left[{\hat{\theta }}_{d}\left(k\right)-{\hat{\theta }}_{0}\left(k\right)\right]}^{2}\right\}}^{1/2}\text{.} \end{array}$$

The following results are given. Tables 1–3 reveal the true value, estimated value, deviation, and root mean square of parameters under different samples.

From the results of deviation and root mean square, it can be seen that even in the case of small samples (*n* = 30), the deviation value is acceptable because more than 80% of the deviation value is less than 0.05, that is, the effective value is about 95%. In terms of root mean square, with the increase of sample size, the root mean square of *σ*_u_ and *β*_0_ decreases uniformly, indicating that the sample size has an impact on the estimation results. To sum up, all the results can show that Bayesian estimation is also close to the real value in the case of small samples, which is consistent with the theoretical results.

## 4. Results and Analysis

### 4.1. Relationship between Students' Learning Adaptation and Mental Health in Information-Based Teaching Environment

Similar to the definition of mental health, different researchers have different opinions on the definition of mental health standards. Maslow believes that a person with the personality characteristics of self-expression is a person with mental health. Drawing on the achievements of researchers at home and abroad, this paper summarizes six standards of mental health: a correct understanding of reality; self-knowledge, self-esteem, and self-acceptance;self-regulation ability [13, 14]; the ability to establish close relationships with people; stability and coordination of lattice structure; and life enthusiasm and work efficiency [15].

Adaptability has always been considered to be closely related to the level of mental health. Kusuma et al. even believe that adaptation to life is one of the constituent elements of mental health [16]. Learning adaptation will not only have a direct impact on students' academic performance but also affect students' psychological development and mental health level. Research shows that there is a significant positive correlation between learning adaptability and mental health. The mental health level of students with high learning adaptability is significantly better than that of students with low learning adaptability [17, 18].

### 4.2. Research Methods

408 students and junior middle school students from the two places were randomly selected to investigate the students' learning situation under the information-based teaching environment (including the basic situation survey, the students' learning adaptability questionnaire, and the mental health questionnaire under the information-based teaching environment) through the network platform developed by the Department of Educational Technology in the University. All students surf the Internet through the computer room of their school and complete the questionnaire anonymously on the Internet. There are 133 primary school students (21 in grade 2, 59 in grade 3, and 53 in grade 4) and 275 junior middle school students (220 in grade 1 and 55 in grade 2), with an average age of 11.75 years; 214 boys and 194 girls; 210 in Beijing and 198 in Guangdong; 382 Han people and 26 ethnic minorities; 227 only children and 181 non-only children; father's education level: 4.9% in primary school, 50.5% in middle school, 32.6% in university, and 12% in master's degree or above; and mother's education level: 8.6% in primary school, 47.1% in middle school, 32.8% in university, and 11.5% in master's degree or above.

#### 4.2.1. Research Tools

Based on the self-regulated learning theory, we propose that students' learning adaptation in the information-based teaching environment includes five dimensions: learning motivation, information acquisition methods, metacognitive strategies, knowledge acquisition, and knowledge expansion [19]. Learning motivation refers to the internal motivation that directly promotes students' learning; information acquisition means the ability to obtain learning resources through information technology; metacognitive strategy refers to the strategy of controlling the process of information and monitoring and guiding the cognitive process; knowledge acquisition and knowledge expansion focus on students' ability to understand and apply knowledge at different stages of the learning process [20]. The questionnaire on students' learning adaptability in the information-based teaching environment (initial version) includes 40 questions, including 8 questions on learning motivation, 6 questions on information acquisition, 8 questions on metacognitive strategies, 12 questions on knowledge acquisition, and 6 questions on knowledge expansion. Using a 4-point score, the subjects are required to respond to the degree of conformity between the situation presented by the questionnaire and themselves according to their actual situation in the past week. The degree of conformity is as follows: very inconsistent (1), relatively inconsistent (2), relatively consistent (3), and very consistent (4). The Mplus robust maximum probability method (MLR) was used for confirmatory factor analysis. According to the correction index, delete the questions with higher correction index. The subscales of the final questionnaire are 6 questions of learning motivation dimension, 4 questions of information acquisition method dimension, 5 questions of metacognitive strategy dimension, 6 questions of knowledge acquisition dimension, and 5 questions of knowledge expansion dimension. *χ*^2^ value is 810.01, DF is 289, CFI is 0.94, TLI is 0.94, SRMR is 0.03, and RMSEA (90% CI) is 0.069 (0.063, 0.074). The correlation between each topic and the total score is greater than 0.35, indicating that the topic has a good discrimination. The homogeneity reliability (*α* coefficient) of the total scale is 0.80, and the homogeneity reliability (*α* coefficient) of each subscale is more than 0.82. In short, the self-made questionnaire on students' learning adaptability in the information-based teaching environment has good reliability and validity [21, 22].

#### 4.2.2. Self-Compiled Student Mental Health Questionnaire

Through literature review, expert discussion, and interviews with primary and secondary school students, this paper summarizes five dimensions of primary and secondary school students' mental health: learning, self, society, emotion, and behavior. Learning refers to the ability of self-regulated learning, including the development of attention, critical thinking, and creative thinking; self includes self-concept, self-evaluation, and self-regulation; society mainly investigates interpersonal relationships, including parent-child, teacher-student, and classmate relationships; emotion mainly refers to the ability of emotion regulation [23]; behavior refers to students' behavior problems such as aggression, hyperactivity, and violation of discipline. Accordingly, we have preliminarily formed a student mental health questionnaire under the information-based teaching environment, with a total of 119 questions, which adopts a 5-point score (0–4). Subjects were asked to answer the severity of the questions in the questionnaire within one week according to their physical and psychological conditions. 0 means no, and 4 means serious. The higher the total score of the questionnaire, the more unhealthy the psychology is [24]. The results of exploratory and confirmatory factor analysis were not ideal. After expert discussion, the questionnaire was modified and a 67-question questionnaire was obtained, including 15 questions on learning dimension, 10 questions on self-dimension, 14 questions on social dimension, 13 questions on emotional dimension, and 15 questions on behavioral dimension. 613 pupils and junior middle school students were tested for the second time, and Mplus7 robust maximum probability method (MLR) was used for confirmatory factor analysis. According to the correction index, delete the questions with higher correction index. The subscales of the final questionnaire are 9 questions of learning dimension, 8 questions of self-dimension, 8 questions of social dimension, 7 questions of emotional dimension, and 15 questions of behavior dimension. *χ*^2^ value is 1242.79, DF is 726, CFI is 0.91, TLI is 0.90, SRMR is 0.05, and RMSEA (90% CI) is 0.034 (0.031, 0.037). The discrimination of the questions is good, and the correlation between each question and the total score is greater than 0.50. The homogeneity reliability (*α* coefficient) of the total scale is 0.96, and the homogeneity reliability (*α* coefficient) of each subscale is more than 0.75. In short, the self-made student mental health questionnaire has good reliability and validity and meets the requirements of psychometrics. Considering the intersection between the learning dimension and learning adaptability in the mental health questionnaire, we removed the learning dimension when analyzing the relationship between learning adaptability and mental health [25].

### 4.3. Result Analysis

Mplus7.0 software and SPSS16.0 software programs were used for data processing and statistical analysis. Using potential profile analysis, this paper discusses the potential categories of students' learning adaptation in the information-based teaching environment composed of five dimensions. Analysis of variance was used to explore the differences of students with different learning adaptation categories in each dimension and total score of mental health.

#### 4.3.1. Descriptive Statistics of Students' Learning Adaptability and Mental Health

The descriptive statistical results are shown in Table 4. The analysis shows that there is a positive correlation between the dimensions and total scores of the learning adaptability questionnaire and the dimensions and total scores of the mental health questionnaire. There is a negative correlation between the dimensions and total scores of the learning adaptability questionnaire and the dimensions and total scores of mental health, and ps < 0.01. In addition, the average scores of each dimension and total score of the learning adaptability questionnaire are greater than 3 points. The highest and lowest dimensions are knowledge acquisition dimension (3.370) and knowledge expansion dimension (3.122), respectively. The scores of each dimension and total score of mental health questionnaire are mainly below 0.5, and the highest and lowest dimensions are social dimension (0.435) and emotional dimension (0.359), respectively.

#### 4.3.2. Potential Profile Analysis of Students' Learning Adaptability

Taking the scores of students in the five dimensions of learning adaptability questionnaire (learning motivation, information acquisition methods, metacognitive strategies, knowledge acquisition, and knowledge expansion) as explicit variables, the potential profile model is established. The fitting indexes of potential profile models with different categories are shown in Table 5.

It is found that the AIC, BIC, and AIBC indexes of the model decrease gradually with the increase of the number of categories. The change range of the three indicators is divided by the number of categories “4.” The change range of the indicators of the first three classification models is large, and the change range of the indicators of the latter three types of models tends to be flat, indicating that with the increase of the number of model classifications, the optimization degree of the latter model gradually decreases compared with the former model. In addition, the entropy value of all category models is greater than 0.94, showing a good degree of model fitting, and the model with the number of categories from 2 to 4 is better (category 2: 0.989; category 3: 0.957; category 4: 0.979). From the perspective of LMRT, the LMRT of the models with four classification numbers from category 2 to category 5 reached a significant level (ps < 0.01). Considering the above fitting indexes and referring to the simplicity and actual situation of the model, four types of models are finally selected as our potential profile analysis model.  Table 6 shows the distribution of the number of people in the four potential categories measured by the learning adaptability questionnaire and the *Z* scores of the corresponding categories in each dimension and total score of the learning adaptability questionnaire.

Among all categories of people, category 1 has the least number, accounting for only 4.2% of the total number, followed by category 2 (7.6%), and categories 3 and 4 account for a large proportion, accounting for 42.9% and 45.3%, respectively.  Figure 6 describes the average scores of the four categories of people in each dimension and total score of the learning adaptability questionnaire.

As shown in the figure, the distribution of the four categories in each dimension and total score is relatively consistent, without too much fluctuation. The first group has the lowest score in all dimensions and total scores and is named “maladjustment group”; the second group was named “troubled group”; the score of the third year group is second only to the fourth group, which is in the middle of the population and is named “marginal adaptation group”; the score of group 4 is the highest in all dimensions and total scores, indicating the best learning adaptability. It is named “good adaptation group.”

Further analysis of variance on the scores and total scores of different categories of people in each dimension of the learning adaptability questionnaire found that there were significant differences in the scores and total scores of each dimension among the four categories (ps < 0.01), which also verified the effectiveness of the four-category model of potential profile analysis from another side. In order to explore the differences in demographic information among the four groups, we counted the distribution proportion of the four groups in terms of “gender,” “whether they are the only child,” “ethnicity,” “father's education level,” and “mother's education level” (Table 7) and conducted a chi square test.

The results showed that there were significant differences in the proportion of categories in the variables of “whether they are the only child,” “father's education level,” and “mother's education level” (ps < 0.01), but there were no significant differences in the proportion of categories in the variables of “gender” (*P*=0.057) and “ethnicity” (*P*=0.604). Further analysis of the variables with significant chi square test shows that in the category proportion composition of the variable “whether it is an only child,” the proportion of “only child” and “not only child” in the first group (“maladaptive group”) and the fourth group (“good adaptation group”) is quite different, and the proportion of “only child” is significantly higher than that of “not only child.” In terms of the category proportion composition of the variable “father's education level,” we found that the proportion of fathers with higher education (graduate and above) in category 1 (“maladjustment group”) and category 4 (“good adaptation group”) was significantly higher than that in category 2 (“troubled group”) and category 3 (“marginal adaptation group”). But at the same time, it is interesting to note that there is an obvious “average” trend in the proportion of fathers' education level in the first group (“maladjustment group”), and the proportion of fathers with “primary school” education level in this group is significantly higher than that in the last three groups. Similarly, in terms of the category proportion of the variable “mother's education level,” the proportion of mothers with higher education (graduate students and above) in category 1 (“maladjustment group”) and category 4 (“good adaptation group”) is significantly higher than that in category 2 (“troubled group”) and category 3 (“marginal adaptation group”). Generally speaking, the “maladjustment group” and “good adaptation group” are more likely to be the only child, and the educational level of their parents is mostly highly educated (graduate students and above), but at the same time, compared with the “good adaptation group,” the proportion of their parents with “primary school” academic experience is also higher.

#### 4.3.3. Differences in Mental Health of Students with Different Types of Learning Adaptation

In order to explore the differences in the scores of various dimensions and total scores of mental health among different categories of students, one-way ANOVA was carried out. The results showed that there were significant differences in the scores of all dimensions and total scores of mental health among different categories of students (ps < 0.01). The posttest found that there were significant differences in the scores and total scores of each dimension between group 2 (“troubled group”) and the group 4 (“good adaptation group”) and between group 3 (“marginal adaptation group”) and group 4 (“good adaptation group”) (ps < 0.01). At the same time, except for the self-dimension, there were significant differences in the scores and total scores of other dimensions between the first group (“maladaptive group”) and the second group (“troubled group”) (*P* social, behavioral and total scores <0.05, *P* emotional <0.01). In addition to self and behavior dimensions, there were also significant differences between group 2 (“troubled group”) and group 3 (“marginal adaptation group”) (*P* social <0.01, *P* emotional and total score <0.05 “(*P* social, behavioral and total scores <0.05, *P* emotional <0.01)” and “(*P* social <0.01, *P* emotional and total score <0.05)” for correctness.” In general, the mental health level of group 2 (“troubled group”) is the worst, and that of group 4 (“well adapted group”) is the best. Comparing the scores of all dimensions and total scores of various groups in the learning adaptability questionnaire, it can be found that when the learning adaptability level is in the middle, the mental health status is poor, while when the learning adaptability is in the two poles (best and worst), the mental health level is better.

### 4.4. Discussion

This study found that there were significant differences in the scores of all dimensions and total scores of mental health among students of different potential categories. The mental health level of the troubled group was the worst, and the mental health level of the well adapted group was the best. When students are at the intermediate level of learning adaptability, their mental health is poor, while when students' learning adaptability is at the two poles (best and worst), their mental health is better. Specifically, when students encounter difficulties in learning adaptation and marginal adaptation, they will feel the greatest learning pressure, which will affect students' self-identity, social communication, and emotional stability and increase the probability of students' problem behavior. When students are extremely unfit for the information-based learning process, they will avoid and maintain themselves. On the contrary, they will have a better mental health level as well as become well adapted students. In the above, we found that the proportion of only child students who are not well educated is higher than that of their parents. This kind of family often has good material conditions and loose family atmosphere, which will also form a protective mechanism for students' mental health, making students have good self-acceptance ability and good mental health level.

## 5. Conclusion and Discussion

Through the potential profile analysis, we find that under the information-based teaching environment, primary and secondary school students can be divided into four subgroups according to learning adaptation: non-adaptation group, distress group, marginal adaptation group, and good adaptation group. There are significant differences in the scores and total scores of all dimensions of learning adaptation (learning motivation, information acquisition methods, metacognitive strategies, knowledge acquisition, and knowledge expansion) among the students of the four groups, showing the gradual rise of adaptation level, which shows that this objective classification method is accurate and effective. The study also found that the proportion of only children is higher among well adapted and maladaptive students, and the educational level of their parents is mostly highly educated (graduate students and above), revealing that only children and students with highly educated parents are prone to polarization in learning adaptability. Among the four types of students, 45.3% are in the good adaptation group and 42.9% are in the marginal adaptation group, which is consistent with our observation. It shows that most students can better deal with the informatization of teaching and learning tools and will try to interact with technology to complete the learning process. These students have high learning motivation, can effectively use various learning strategies, can obtain learning resources, and can understand and use knowledge, so as to achieve better learning results. The study also found that 7.6% of students are in the troubled group and 4.2% are in the maladjustment group. Although the number of these two types of students is small, they are at a low level in all aspects of learning adaptation, which may lead to their poor learning. In practical work, teachers can use the potential profile analysis method to identify students with learning maladjustment and build a more adaptive learning environment to guide and adjust these students from the aspects of motivation, strategy, information acquisition mode, knowledge mastery, and application, so as to help them get rid of learning difficulties.

## Figures and Tables

**Figure 1:** Common puzzles of college students.

**Figure 2:** Straight line diagram under different quantiles (beta = 0.05).

**Figure 3:** Straight line diagram under different quantiles (beta = 0.25).

**Figure 4:** Straight line diagram under different quantiles (beta = 0.75).

**Figure 5:** Straight line diagram under different quantiles (beta = 0.95).

**Figure 6:** Distribution of scores of various groups of others on the learning adaptability questionnaire.

**Table 1:** *n* = 30.

Parameters	True value	Estimated value	Root mean square	Deviation
*β*_0_	0.5	0.560	0.050	0.060
*β*_1_	0.7	0.657	0.041	0.025
*β*_2_	0.7	0.734	0.042	0.034
*β*_3_	0.7	0.667	0.049	0.033
*β*_4_	0.7	0.742	0.042	0.042
*σ*_u_	0.8	0.950	0.162	0.150

**Table 2:** *n* = 50.

Parameters	True value	Estimated value	Root mean square	Deviation
*β*_0_	0.5	0.540	0.032	0.040
*β*_1_	0.7	0.680	0.042	0.020
*β*_2_	0.7	0.730	0.039	0.030
*β*_3_	0.7	0.670	0.042	0.030
*β*_4_	0.7	0.722	0.040	0.022
*σ*_u_	0.8	0.860	0.086	0.060

**Table 3:** *n* = 100.

Parameters	True value	Estimated value	Root mean square	Deviation
*β*_0_	0.5	0.520	0.025	0.020
*β*_1_	0.7	0.669	0.044	0.031
*β*_2_	0.7	0.672	0.036	0.028
*β*_3_	0.7	0.680	0.032	0.020
*β*_4_	0.7	0.673	0.037	0.027
*σ*_u_	0.8	0.792	0.007	0.008

**Table 4:** Descriptive statistics and correlation of main variables.

	Dimension and total score	Learning adaptability						Mental health				
		1.1	1.2	1.3	1.4	1.5	1.6	2.1	2.2	2.3	2.4	2.5
1 learning adaptability	1.1 motivation	1										
	1.2 way	0.870^*∗∗*^	1									
	1.3 policy	0.837^*∗∗*^	0.902^*∗∗*^	1								
	1.4 get	0.897^*∗∗*^	0.884^*∗∗*^	0.911^*∗∗*^	1							
	1.5 expand	0.849^*∗∗*^	0.833^*∗∗*^	0855^*∗∗*^	0.854^*∗∗*^	1						
	1.6 total score	0955^*∗∗*^	0.941^*∗∗*^	0.959^*∗∗*^	0.962^*∗∗*^	0.923^*∗∗*^	1					

2 mental health	2.1 self	−0.302^*∗∗*^	−0.244^*∗∗*^	−0.263^*∗∗*^	−0.266^*∗∗*^	−0.242^*∗∗*^	−0.280^*∗∗*^	1				
	2.2 society	−0.0.299^*∗∗*^	−0.240^*∗∗*^	−0241^*∗∗*^	−0.280^*∗∗*^	−0.228^*∗∗*^	−0.275^*∗∗*^	0.830^*∗∗*^	1			
	2.3 emotional	−0.302^*∗∗*^	−0.259^*∗∗*^	−0.258^*∗∗*^	−0.286^*∗∗*^	−0.254^*∗∗*^	−0.289^*∗∗*^	0.788^*∗∗*^	0.829^*∗∗*^	1		
	2.4 behavior	−0.300^*∗∗*^	−0.227^*∗∗*^	−0.251^*∗∗*^	−0.270^*∗∗*^	−0.215^*∗∗*^	−0.270^*∗∗*^	0821^*∗∗*^	0.812^*∗*^	0.798^*∗∗*^	1	
	2.5 total score	−0324^*∗∗*^	−0 261^*∗*^	−0.273^*∗∗*^	−0.297^*∗∗*^	−0.253^*∗∗*^	−0.300^*∗∗*^	0934^*∗∗*^	0.936^*∗∗*^	0.915^*∗∗*^	0.923^*∗*^	1
	Average	3.203	3.291	3.289	3.370	3.122	3.256	0.435	0.359	0.398	0.407	0.400
	Deviation	0.744	0.765	0.720	0.736	0.692	0.694	0.584	0.529	0.542	0.494	0.498

^*∗*^ *P* < 0.05; ^*∗∗*^*P* < 0.01.

**Table 5:** Fitting index of learning adaptation potential profile model.

	1 kind	2 kind	3 kind	4 kind	5 kind	6 kind
AIC	4526.822	3278.074	2115.758	1618.085	1398.033	1376.636
BIC	4566.934	3342.254	2204.006	1730.401	1534.416	1537.086
AIBC	4535.203	3291.483	2134.196	1641.552	1426.529 1	410.160
Entropy		0.989	0.957	0.979	0.948	0.953
LMRT		0.000^*∗∗*^	0.000^*∗∗*^	0.000^*∗∗*^	0.018^*∗*^	0.101

^*∗*^ *P* < 0.05; ^*∗∗*^*P* < 0.01.

**Table 6:** Characteristic distribution of four category models.

Classification	*n*	%	*Z* score for the learning adaptation questionnaire					
			Academic motivation	Information acquisition method	Metacognitive strategy	Knowledge to obtain	Knowledge extension	Total points (TPs)
1	17	4.167	−2.749	−2.897	−3.031	−3.152	−2.931	−3.111
2	31	7.598	−1.588	−1.599	−1.428	−1.540	−1.137	−1.544
3	175	42.892	−0.301	−0.273	−0.308	−0.211	−0.293	−0.290
4	185	45.343	0.803	0.793	0.809	0.747	0.737	0.819

**Table 7:** Proportion distribution of the number of people in four groups.

		Category 1 “unfit group” (%)	Category 2 “troubled group” (%)	Category 3 “edge adaptation group” (%)	Category 4 “well adapted group” (%)
Sex	Male	76.5	64.5	47.4	53.0
	Female	23.5	35.5	52.6	47.0

Only child	Yes	82.4	45.2	42.9	67.0
	No	7.6	54.8	57.1	67.0

Ethnicity	Han	100.0	90.3	93.1	94.1
	Minority	0	9.7	6.9	5.9

Father's level of education	Primary school	23.5	16.1	8.6	4.3
	Middle school	23.5	48.4	58.3	39.5
	Undergraduate course	35.3	32.3	29.1	35.7
	Graduate student or above	17.6	3.2	4.0	20.5

Education level of the mother	Primary school	17.6	19.4	20.6	28.6
	Middle school	41.2	45.2	44.6	36.2
	Undergraduate course	29.4	32.3	31.4	24.6
	Graduate student or above	11.8	3.2	3.4	220.5

## Data Availability

The labeled dataset used to support the findings of this study is available from the corresponding author upon request.
